# Vehicle Image Detection Method Using Deep Learning in UAV Video

**DOI:** 10.1155/2022/8202535

**Published:** 2022-02-08

**Authors:** Xiangqian Wang

**Affiliations:** School of Information on Engineering, Pingdingshan University, Pingdingshan, Henan, 467000, China

## Abstract

Traditional machine learning algorithms are susceptible to objective factors such as video quality and weather environment in the vehicle detection of Unmanned Aerial Vehicle (UAV) videos, resulting in poor detection results. A vehicle image detection method using deep learning in UAV video is proposed. The algorithm in this paper treats surveillance video as many frames of images for vehicle detection in the image. First, perform HSV (Hue-Saturation-Value) spatial brightness translation operation on the original sample to increase the adaptability to different light conditions and sample diversity. Then, the Single Shot MultiBox Detector (SSD) model framework is used as the basis for vehicle detection. In order to obtain a better feature extraction effect, focus loss is added to the basic SSD for optimization. Finally, the trained network model is used to analyze the UAV video, and the detection performance is analyzed experimentally. The results show that the vehicle detection rate of this algorithm has reached 96.49%. It can ensure that the vehicle is accurately detected from the drone video.

## 1. Introduction

As the pace of urbanization in our country continues to accelerate, the number of roads and family cars in our cities is increasing, and road traffic pressure is increasing day by day. The research of intelligent transportation system is very important to ensure the smoothness and safety of roads [1, 2]. Intelligent transportation system uses information technology, such as image recognition, computer vision, etc. to realize more intelligent and automated road transportation system. It improves the throughput capacity of the road area and greatly facilitates the dispatch of the traffic management department. However, real-time acquisition of road traffic information is the basis for the realization of an intelligent transportation system. How to obtain high-quality road vehicle information has become an urgent problem to be solved.

At present, the collection methods of vehicle information mainly include loop coil detection, infrared detection and intelligent video surveillance detection [3–5]. Among them, the loop coil detection work is stable, the detection accuracy is high, and the traffic information can be counted. It is easy to install and set up, and is mostly used in areas such as traffic toll crossings and parking lots. Infrared detection mainly uses light-emitting diodes to detect vehicle speed, with high detection sensitivity. But it is easily affected by the environment, such as temperature, humidity, etc., resulting in low detection accuracy and low robustness. With the development of technologies such as image recognition and computer vision, intelligent video surveillance and detection has taken up an increasingly important position in traffic information collection. Intelligent video surveillance detection uses a camera set up at a traffic intersection to perform target analysis on the camera monitoring area to obtain unstructured information of the target in the video. The traffic monitoring video contains a wealth of information and is an important data source for intelligent traffic monitoring systems [6]. However, the data resources acquired by fixed cameras are limited. With the development of drone technology, it has begun to be widely used in traffic monitoring, with rich data types and efficient data acquisition. But how to detect the vehicle from the massive data is the difficulty of the research [7, 8].

At present, there have been many researches on vehicle identification in surveillance video. Reference [9] proposed an automatic detection method for smoke vehicles in traffic surveillance videos based on vehicle rear detection and multi-feature fusion. Using the Vibe background subtraction algorithm to detect foreground objects and remove non-vehicle objects according to the rules. An improved integral projection method is used to detect the rear of the vehicle to obtain the key area behind the rear of the vehicle. Effectively improve the accuracy of road safety early warning. Reference [10] proposed a smoke vehicle detection method by learning spatio-temporal representation from image sequences. The motion detection algorithm is used to obtain the tail of the vehicle that needs to be identified. And using time multi-layer perception or long short-term memory network to effectively train the smoke vehicle recognition model, which effectively improves the recognition accuracy. Reference [11] proposed a preprocessing framework with virtual single-layer sequences in traffic video surveillance. By fusing the effective element estimation module and the dynamic multi-stage parallel video image processing module, the robustness and effectiveness of vehicle detection in the video are improved.

With the rapid development of computer technology, machine learning algorithms have also been widely used in the field of image recognition. Reference [12] compares several commonly used video vehicle recognition methods including deep learning models and computer vision methods. The average accuracy, the semantics of recognizing vehicles, and the robustness of recognition when applied to data sets containing images with different lighting conditions are used to compare detection accuracy. The results show that the proposed deep learning method has better recognition performance. Reference [13] proposed a driver warning and collision avoidance system based on vehicle trajectory characteristics and long- and short-term memory neural network. By judging the video behavior of vehicles, road safety is effectively improved. However, the initial detection performance of the vehicle in the video still needs to be optimized. Reference [14] proposed a new type of hybrid artificial neural network and a mobile vehicle detection system based on the opposing gravity search optimization algorithm. Used to detect moving vehicles in traffic scenes to achieve effective traffic video surveillance. Optimizing the selection weights through the opposing gravity search optimization algorithm, effectively improving the recognition accuracy and speed of the artificial neural network. Reference [15] proposed a region-based Convolutional Neural Network (CNN) in vehicle detection algorithm. The rapid aggregation of road traffic data is effectively realized to improve traffic automation management. However, the above method is limited to the transmission image of the fixed camera for traffic video, and the flexibility is poor. Compared with ordinary video surveillance scenes, the video collected by drones has the advantages of wide surveillance range, less target occlusion, and more macroscopic traffic information provided. However, most existing machine learning methods are difficult to process real-time and massive drone video data. For this reason, a vehicle image detection method using deep learning in UAV video is proposed. The innovations of the proposed method are summarized as follows:

1. Because a variety of different models, different appearances, and vehicle videos shot from different angles are collected from multiple video scenes. Light has a great influence on video recognition. The proposed method performs a spatial brightness translation operation on the original sample. To increase the adaptability of the classifier to different light conditions and sample diversity.
2. In order to obtain a better feature extraction effect, the proposed method adds focus loss to the basic SSD for optimization to improve the detection accuracy.

## 2. UAV Video Characteristics Analysis

The video data used was hovered 50 meters directly above the road by the DJI phantom3 professional drone, and the camera lens was shot at −90°. The video resolution is 3840 × 2160. Video characteristics affect the choice of vehicle detection methods. Compared with ground-based fixed video, UAV video is mainly different in the following six aspects:

1. Traffic information is more comprehensive, which is more valuable for application and research. From the UAV video, not only traffic information such as traffic flow and speed can be obtained, but also the traffic density of the road section and the accurate vehicle trajectory can be directly obtained [16]. It has important value in the study of traffic flow theory, driving behavior, car following (lane changing) and other traffic theories.
2. There are more vehicles in the detection range, the smaller the vehicle size, and the greater the difficulty of detection. The UAV video image can contain hundreds of vehicles, so the vehicle size is small and the feature information is less.
3. The video coverage is wider and the interference information is more. Under the premise of being able to detect vehicles, the UAV video range can reach up to several hundred meters. In addition to the concerned vehicle information in the image, there is also a large amount of invalid information. For example, buildings, street lights, signs and markings, motorcycles, etc.
4. Different vehicle imaging has different vehicle detection methods. Usually, a fixed ground camera shoots the front or back of the vehicle. The drone shoots the top of the vehicle and uses the line characteristics to detect the vehicle in the fixed video. UAV video uses other methods.
5. Video jitter is more obvious. Although the camera is installed on the drone's airborne gimbal, the drone is affected by the wind during the hovering flight, and the captured video image still exhibits irregular jitter. This increases the difficulty of accurately detecting vehicles [17].
6. Due to the limitations of the drone's flight capability and endurance, it is usually only possible to obtain traffic videos in better weather conditions. The effective shooting time does not exceed 20 minutes.

The experimental data is a traffic video taken by a drone in a certain place in Zhengzhou in 2020. The video frame rate is 30 frames per second, and the video resolution is 1920 × 1080. Video 01 was shot at a straight intersection. Video 02 was shot at a T-junction. Video 03 was shot on an elevated section. The first frame of the experimental data is shown in Figure 1. And the detailed information of the experimental data is shown in Table 1.

## 3. Algorithm Design

### 3.1. Design Ideas of Vehicle Classifier

To achieve vehicle detection from the perspective of deep learning, use CNN method in deep learning to design a vehicle detector. The vehicle detector is realized by detecting whether the object in each detection frame is a vehicle. Therefore, it is necessary to design a vehicle classifier with improved CNN to realize the two-class classification of cars and non-cars. The process of training and testing the classifier model is shown in Figure 2.

First carry out a preprocessing operation on the training samples. Then put the training samples and corresponding labels into CNN for training, and get an improved CNN model. Then the test samples are also preprocessed, and the prediction results of the model are obtained by improving the CNN model. The prediction result is compared with the test sample label, and the final test result is obtained.

### 3.2. Dataset Preprocessing

#### 3.2.1. Sample Collection

The size of 50 × 50 is selected as the input image size of the trained classifier, which is also the size of the vehicle detection frame in the actual video. For images whose sample size does not meet the requirements, the original samples that meet the requirements are obtained through cropping and scaling operations.

Because there is no vehicle sample set that includes different models and different angles. In multiple videos and many pictures, 2503 positive samples and 2,698 negative samples are collected to form a relatively complete vehicle classification data set. The pictures in the positive sample set include vehicles of different brands and types, and the angles at which they are taken are also different. The light conditions and background of each sample are also different, which fully guarantees the diversity of positive samples. If the classifier can identify these types of vehicles with different backgrounds, it is enough to show that the proposed classifier has strong adaptability [18, 19]. The negative sample set includes various background scenes without vehicles that may appear around the road. For example, there may be road signs, tree shades, pedestrians, trees, etc., which are also sufficiently diverse [20, 21].

#### 3.2.2. Data Preprocessing

In order to enhance the adaptability of the classifier to different lighting environments and in the shade, the original data set is preprocessed in the HSV space. In the HSV color space, the V value represents the brightness, which is the brightness of the color, and it is also expressed as a percentage. Its value ranges from 0%, which means completely black, to 100%, which means completely bright. Therefore, the brightness can roughly indicate the brightness of the entire scene, and the brightness of the scene can be changed by the brightness shift operation. Shift the average V value of each original picture to 20%, 30%, 40%, 50%, 60% (because it is too dark at 20%, and the scene is too bright at 70%). While keeping the H value and S value unchanged, the new V value corresponding to each point is:

(1) $$\begin{array}{c} V_{\text{new}}\left(a,b\right)=\frac{V_{\text{old}}\left(a,b\right)\times {\bar{V}}_{\text{new}}}{{\bar{V}}_{\text{old}}}, \end{array}$$

where *V*_new_(*a*, *b*), *V*_old_(*a*, *b*), ${\bar{V}}_{\text{new}}$, ${\bar{V}}_{\text{old}}$ represent the new lightness value, the old lightness value, the new lightness mean value and the old lightness mean value, respectively.

Through the above processing, a sample set covering multiple different brightness values is obtained. The number of positive and negative samples in the sample set has increased to 15,426 and 17,071 respectively. Before processing, first convert the image from RGB (Red-Green-Blue) to HSV space. After processing, all pictures need to be converted back to RGB space.

After that, all the samples processed above are grayed out. Using *R*(*a*, *b*), *G*(*a*, *b*) and *B*(*a*, *b*) to denote the components of the *R*, *G*, and *B* channels of the pixel at position (*a*, *b*), respectively. Then the gray value of the corresponding point:

(2) $$\begin{array}{c} G\left(a,b\right)=0.2989\times R\left(a,b\right)+0.5870\times G\left(a,b\right)+0.1140\times B\left(a,b\right). \end{array}$$

After grayscale, the grayscale value range of the grayscale image is [0, 255]. Finally, perform a simple normalization operation on the grayscale image data to obtain the input layer sample data:

(3) $$\begin{array}{c} I\left(a,b\right)=\frac{G\left(a,b\right)}{255}. \end{array}$$

In summary, the preprocessing process of the original image is shown in Figure 3.

### 3.3. SSD Target Detection

The SSD network uses the classic network VGG as the basic network. Adding auxiliary structure after the basic network produces a detection with the following main characteristics.

The SSD network uses multi-scale feature map detection. The network adds the convolutional feature layer to the end of the extreme base. The size of these layers gradually decreases, and multiple scale detections are predicted values [22, 23]. The detected convolution model is different for each feature layer. Each feature layer (or optional existing feature layer of the base network) can use a set of convolution filters to generate a fixed set of predictions. For the feature layer of size *m* × *n* with *d* channels, use the 3 × 3 × *d* convolution kernel convolution operation to generate the score of category or the coordinate offset relative to the default box. At each *m* × *n* size position where the convolution kernel operation is applied, an output value is generated. The output value of the bounding box offset is measured relative to the default box, and the default box position is relative to the feature map. The core of the SSD algorithm is to use both high-level feature maps and low-level feature maps for detection. The feature maps of different layers are used to imitate the detection of objects at different scales. The default candidate box refers to a series of fixed-size bounding boxes on each small grid of the feature map, as shown in Figure 4.

Assume that there are *k* default candidate boxes for each cell in each feature map. Each default candidate box needs to predict *p* category scores and 4 coordinate information. If the size of a feature map is *m* × *n*, then each feature map has *m* × *n* × *k* × (*p*+4) outputs. The meaning of these outputs is that a 3 × 3 convolution kernel is used, and the number of convolution kernels when convolving the feature map of this layer contains two parts. The first part of the quantity *m* × *n* × *k* × *p* is the output of confidence, which represents the confidence of each default candidate box, that is, the probability of the category. The second part 4 × *m* × *n* × *k* is the output of the coordinate position, which represents the coordinate of each default candidate box after returning.

In training, another concept is a priori candidate box. Refers to the default alternative box selected in practice. During training, a complete picture is input to the network to obtain several feature maps [24]. For positive sample training, it is necessary to first match the prior candidate box with the correctly labeled candidate box. A successful match indicates that the a priori candidate box is the target to be detected, but there is still a certain gap from the complete target. The purpose of training is to ensure the classification confidence of the default candidate box while returning the prior candidate box to the correctly labeled bounding box as much as possible. For example, suppose there are 2 correctly labeled bounding boxes in a training sample. There are totally 8732 default candidate frames obtained in all feature maps. Then there may be 10 and 20 a priori candidate boxes that can be matched with the two correctly labeled bounding boxes respectively. The training loss includes positioning loss and regression loss.

Experiments have shown that the greater the number of default candidate box shapes, the better the final effect. The default candidate box used here is the same as the candidate box in Faster R–CNN. The difference is that the candidate box in Faster R–CNN is only used in the last convolutional layer, but in SSD, the default candidate box is applied to multiple different feature maps. The size and aspect ratio of the default candidate box are determined by certain calculations. Assuming that *g* feature maps are used for prediction, the size of the default candidate box for each feature map is calculated as follows:

(4) $$\begin{array}{c} s_{k}=s_{\min}+\frac{s_{\max}-s_{\min}}{g-1}\left(k-1\right),\;k\in \left[1,g\right], \end{array}$$

where, *s*_min_=0.2 indicates that the size of the bottom layer is 0.2. *s*_max_=0.9 indicates that the size of the highest layer is 0.9.

For the aspect ratio, it is represented by *β*_*r*_. There are five aspect ratios, namely *β*_*r*_={1,2,3, 1/2, 1/3}. Therefore, the width of each default candidate box is calculated as $w_{k}^{\beta }=s_{k}\sqrt{\beta_{r}}$. The calculation formula for height is $h_{k}^{\beta }=s_{k}\sqrt{\beta_{r}}$. In addition, when the aspect ratio is 1, specify the size as $s_{k}=\sqrt{s_{k}s_{k+1}}$ additionally. That is, there are a total of 6 different default candidate boxes.

The center position of each default candidate box on the feature map is set to (*a*+0.5/|*f*_*k*_|, *b*+0.5/|*f*_*k*_|). Where |*f*_*k*_| represents the size of the *k* th feature map. The default frame coordinates captured by *a*, *b* ∈ (0, |*f*_*k*_|) make it always within [0, 1]. In fact, the distribution of default boxes can be designed to best fit a particular database.

By combining the predictions of all default boxes of different sizes and aspect ratios of many feature maps at all positions, a diversified set of predictions can be obtained, covering various input object sizes and shapes [25].

After the default candidate box is matched with the correctly labeled target box, it can be known that most of the default candidate boxes are negative samples, especially when the number of possible default selected boxes is large. This leads to a serious imbalance of positive and negative samples during training. The SSD algorithm is sorted according to the highest confidence of each default candidate box. And choosing those candidate boxes with high confidence so that the ratio between positive and negative samples is at most 3 : 1, instead of using all negative samples. After such processing, the optimization speed of the training process is faster and more stable.

In order to make the model more robust to the size and shape of various input objects, each training image is randomly sampled by one of three methods. (1) Using the entire original image as input. (2) Sampling a small fragment to make the object's smallest Intersection over Union (IoU) overlap of 0.1, 0.3, 0.5, 0.7, or 0.9. (3) Randomly sample a segment. The size of each sample segment is between 0.1 and 1 times the size of the original image, and the aspect ratio is between 0.5 and 2. If the correctly labeled target frame is in the sample segment, the overlapped part is retained. After the above sampling steps, the size of each sampling slice is adjusted to a fixed size and flipped horizontally with a probability of 0.5.

The commonly used objective loss function for multi-classification tasks is cross-entropy loss. Assuming that there are *n* samples in the task and the classification target has *C* class, the cross entropy CE is defined as follows:

(5) $$\begin{array}{c} \text{CE}=\frac{1}{n}\overset{n}{\underset{i=1}{\sum }}\overset{C}{\underset{j=1}{\sum }}-y_{j}^{\left(i\right)}lb\left(\hat{f}{\left(x^{\left(i\right)}\right)}_{j}\right), \end{array}$$

where, $\hat{f}\left(x\right)$ represents the predicted class probability. *y* is the one-hot vector of the actual category. The cross entropy function itself treats all types of objects equally. When encountering category imbalance phenomenon, it is easy to cause prediction deviation, and it is impossible to strengthen training on difficult-to-separate samples. In view of the category imbalance phenomenon, a weighting factor *α* can be introduced for different categories to weaken the influence of a large number of categories on the loss value:

(6) $$\begin{array}{c} \text{CE}=\frac{1}{n}\overset{n}{\underset{i=1}{\sum }}\overset{C}{\underset{j=1}{\sum }}-\alpha_{j}y_{j}^{\left(i\right)}lb\left(\hat{f}{\left(x^{\left(i\right)}\right)}_{j}\right). \end{array}$$

Aiming at the problem of difficult samples, the higher the predicted probability of a sample, the stronger the model's ability to recognize the sample. This sample becomes an easy-to-separate sample, and vice versa, it is a difficult-to-separate sample. Based on the predicted probability, a weighting factor *β* can be introduced to weaken the influence of easily divided samples on the loss value. *β* is defined as follows:

(7) $$\begin{array}{c} \beta_{j}^{\left(i\right)}={\left(1-y_{j}^{\left(i\right)}\right)}^{\gamma }, \end{array}$$

where *γ* is an adjustable hyper parameter. The focus loss FL is defined as:

(8) $$\begin{array}{c} \text{FL}=\frac{1}{n}\overset{n}{\underset{i=1}{\sum }}\overset{C}{\underset{j=1}{\sum }}-\alpha_{j}\beta_{j}^{\left(i\right)}y_{j}^{\left(i\right)}lb\left(\hat{f}{\left(x^{\left(i\right)}\right)}_{j}\right). \end{array}$$

This paper applies the above-defined multi-category focus loss to the SSD model. The values of *α* and *γ* are both 0.75.

The SSD algorithm uses VGG16 as the basic network. First, perform pre-training on the data set, and convert Full Connection Layer (FC) 6 and FC7 into convolutional layers. The parameters are sampled from the FC6 and FC7 layers, and all dropout layers and FC8 layers are deleted. And using Stochastic gradient descent (SGD) to fine-tune the model. For each data set, the learning rate decay strategy is slightly different.

### 3.4. Network Training

Before training, perform image enhancement by performing operations such as horizontal flipping, contrast enhancement, saturation enhancement, and color transformation on all images. All models are implemented using the Tensorflow framework and trained for 400 cycles on the Nvidia1080 graphics card. For the Faster R–CNN model, the images are uniformly scaled to 1280 × 720 input network. The initial learning rate is 0.001. It drops to 1/10 of the previous value every 100 cycles. The gradient update method uses small batch stochastic gradient descent with momentum. The momentum factor is 0.99. For SSD models, the images are uniformly scaled to 500 × 500 input network. The initial learning rate is 0.001. Every 10 cycles it drops to 0.96 times the previous value. The gradient update uses RMSProp optimizer. The momentum factor is 0.99.

## 4. Experiment and Analysis

The hardware operating environment of the experiment is an Intel Core i5-6500 CPU, a notebook computer with a frequency of 3.20 GHz and a memory of 32 GB. The software environment mainly includes Windows 10 system, Visual Studio 2017 development environment and Open CV 3.2.0. Open CV is an open source computer vision library that provides various graphics processing functions. Open CV implements many general algorithms in graphics processing and computer vision. Among them, modules such as 2D features in Open CV, high-level interaction, video image reading and writing, image processing, and target tracking are mainly used. The proposed method is developed independently, and the development language is C++.

### 4.1. Evaluation Index

The goal of vehicle detection is to detect as many vehicles as possible. At the same time, as little as possible misdetection of vehicles occurs. In a real-world vehicle video stream, True Positive Rate (TPR), False Positive Rate (FPR), Average True Positive per Frame (ATP/Frame), Average False Positive per Frame (AFP/Frame), Average False Positive per Vehicle (AFP/Vehicle) and other indicators are evaluated. Among them, the last three index parameters are related to the actual video stream. Therefore, it is only used to evaluate the detection effect of the vehicle detection method in the real scene video stream. The first two parameters are not necessarily related to the video stream, and can also be applied to the training set and test set to evaluate the vehicle classification method.

TPR is the proportion of the number of vehicles *Q*_TP_ correctly detected as TP by the detector or classifier in a video stream segment or sample set to the actual total number of vehicles *Q*_Total_:

(9) $$\begin{array}{c} \text{TPR}=\frac{Q_{\text{TP}}}{Q_{\text{Total}}}. \end{array}$$

FPR is the proportion of the number of targets *Q*_FP_ incorrectly determined as vehicles (FP) by the detector or classifier in all target *Q*_P_ determined as vehicles in a video stream segment or sample set:

(10) $$\begin{array}{c} \text{FPR}=\frac{Q_{\text{FP}}}{Q_{\text{P}}}. \end{array}$$

ATP/Frame is the average number of vehicles correctly detected per frame in a video stream segment:

(11) $$\begin{array}{c} \frac{\text{ATP}}{\text{Frame}}=\frac{Q_{\text{TP}}}{z_{\text{Frames}}}. \end{array}$$

AFP/Frame is the number of vehicles that have been misdetected as non-vehicle targets in each frame in a video stream segment:

(12) $$\begin{array}{c} \frac{\text{AFP}}{\text{Frame}}=\frac{Q_{\text{FP}}}{z_{\text{Frames}}}. \end{array}$$

AFP/Vehicle is the ratio of the number of misdetected targets to the total number of vehicles Ω_Vehicles_ in a traffic video stream segment:

(13) $$\begin{array}{c} \frac{\text{AFP}}{\text{Vehicle}}=\frac{Q_{\text{FP}}}{\Omega_{\text{Vehicles}}}. \end{array}$$

By evaluating the above indicators of the video stream or sample set, the detection performance of a classifier or detector can be evaluated. Based on the above indicators, the higher the TRP, ATP/Frame, and the lower the FPR, AFP/Frame, AFP/Vehicle, the better the performance of vehicle detection method.

### 4.2. Compare the Classification Effects of Different Classifiers

First, compare the classification results of the proposed method with linear discriminant analysis (LDA), support vector machine (SVM) and other shallow classifiers on the test sample set.

It can be seen from Table 2 that among the shallow classifiers, the SVM classifier performs well in many sample sets. The same applies to the test sample set consisting of 3068 test samples. The classification accuracy rate using LDA is only 70.89%. Using the SVM classifier can increase the accuracy by about 19% to 89.11%. The proposed method has undergone 10-fold cross-validation, and finally obtained a relatively stable classification accuracy of 94.92%, which is 5 percentage points higher than the SVM method. This shows that the proposed method has a better classification effect than shallow classifiers in processing two-dimensional data sets. It is more suitable for vehicle detection.

Specifically, the entire test sample set is classified by the proposed method. The results are shown in Table 3.

According to the number of TP, TN, FP, and FN in Table 3, the sensitivity of the proposed method can be obtained: *S*_*n*_=TP/TP+FN=1399/1399+62 × 100%=95.76%; The specificity is: *S*_*P*_=TN/TN+FP=1581/1581+26 × 100%=98.38%; Therefore, the first type of error rate (false positive rate) of the classification model: 1 − *S*_*p*_=1.62% indicates that 1.62% of the real non-vehicle samples were incorrectly judged as vehicle samples. The second type of error rate (false negative rate): 1 − *S*_*n*_=4.24% indicates that among all the vehicle samples, 4.24% of the vehicles were not detected and were misjudged as vehicles.

The detailed classification results of the proposed method and LDA and SVM methods on the test set are shown in Table 4.

It can be seen from Table 4 that in the entire sample set, the TPR of the proposed method is 16.77% and 7.94% higher than that of the LDA and SVM classifiers, respectively. The FPR is 18.03% and 5.27% lower than LDA and SVM, respectively. It shows that under the comprehensive evaluation of these two performance indicators, the proposed method has better detection effect and fewer false detections.

The preprocessing of the original sample will have a greater impact on the later vehicle detection. Therefore, before and after preprocessing, the classification accuracy results of the three methods are shown in Table 5. The second column of data in the table is the classification accuracy of the three methods for the original samples without HSV spatial brightness translation. The third column of data corresponds to the training result after the original sample is subjected to a large brightness shift in the HSV color space.

It can be seen from Table 5 that the classification accuracy of LDA in the two cases is not much different, the difference is only 0.36%. However, the accuracy of SVM and the proposed method under the preprocessing of HSV data is about 5% higher than that of unprocessed data. It can be seen from this that sample training is required for vehicle detection. A richer sample set can significantly improve the classification performance of the classifier.

### 4.3. Performance Comparison of Different Models

In order to demonstrate the detection performance of the proposed model, compare it with reference [9, 11], and [15], and the results are shown in Table 6.

It can be seen from Table 6 that compared with other comparison models, the detection effect of the proposed model is better, and its TPR reaches 96.49%. Reference [9] realizes the automatic detection of smoke vehicles based on multi-feature fusion and improved integral projection method. It can accurately detect vehicles to a certain extent. However, the detection method is relatively traditional, and it is difficult to apply to UAV video data. Therefore, the detected TPR is only 81.92%. Reference [10] uses motion detection algorithms to acquire vehicle information, and uses temporal multi-layer perception or long- and short-term memory networks to train vehicle recognition models. Compared with reference [9], it can effectively improve the recognition accuracy, with a TPR of 88.61%. However, the UAV moves fast and has a lot of video data, so the recognition effect is limited to a certain extent. Reference [15] uses the regional CNN network to achieve vehicle detection, which can quickly aggregate road traffic data, thereby improving automated traffic management. However, it lacks data preprocessing, so the recognition accuracy rate of the proposed method is reduced by 3% to 6%. All the proposed models can achieve better vehicle detection. It uses HSV for data preprocessing, and both deep learning models can complete accurate learning of massive data.

## 5. Conclusion

The accuracy and stability of UAV video vehicle detection is crucial to extracting traffic information. For this reason, a vehicle detection method using deep learning in UAV video is proposed. Based on the HSV spatial brightness translation operation of the original samples, two deep learning models, the improved Faster R–CNN and SSD, are used to detect vehicles in UAV videos. Based on the DJI UAV's shooting video data set for experimental analysis. The results show that the use of HSV for data transformation can enrich the sample set, thereby improving the detection accuracy. The accuracy before and after pretreatment is increased by about 5%. The SSD model of the proposed method processes the data after HSV transformation, and the powerful data learning ability of the model can improve the detection effect. Its vehicle detection rate reached 96.49%. And the SSD model can act on multiple feature maps, and its detection effect is better.

Deep learning technology has shown great potential in target detection, and it is more advantageous for rapid target detection in complex scenes. However, deep learning requires large samples for support, and speed is not an advantage. These two determine the limitations of deep learning in real-time target tracking applications. Therefore, in the future, we will focus on the application of deep learning under small sample training in video target detection, and focus on solving real-time problems.

## Figures and Tables

**Figure 1:** First frame image of experimental data (a) Video 01 (b) Video 02 (c) Video 03.

**Figure 2:** Process of training and testing CNN classifier.

**Figure 3:** Preprocessing process of sample set.

**Figure 4:** The generation of default candidate box (a) Image with GT boxes (b) 8 × 8 characteristic map (c) 4 × 4 characteristic map.

**Table 1:** Details of experimental data.

No.	Length of time	Total frames
01	3 minutes and 35 seconds	5189
02	6 minutes and 12 seconds	12037
03	5 minutes and 49 seconds	10915

**Table 2:** Classification accuracy of different classifiers.

Classifier type	Number of correct tags/total tags	Accuracy rate (%)
LDM	2175/3068	70.89
SVM	2734/3068	89.11
Proposed method	2912/3068	94.92

**Table 3:** The classification effect of the proposed method in the test sample set.

Number	Judged as positive sample	Judged as negative sample	Total
Actual positive sample	1399 (TP)	62 (FN)	1461
Actual negative sample	26 (FP)	1581 (TN)	1607
Total	1425	1643	3068

**Table 4:** Detailed classification results of different methods in the test sample set.

Method	LDA	SVM	Proposed method
Number of positive samples	1461	1461	1461
Number of positive samples detected	1154	1283	1399
Number of negative samples	1607	1607	1607
Number of negative samples detected	1288	1493	1581
TPR (%)	78.99	87.82	95.76
FPR (%)	19.85	7.09	1.82

**Table 5:** Classification accuracy of different methods before and after pretreatment of original samples.

Method	Accuracy rate (%) (Raw data)	Accuracy rate (%) (HSV)
LDA	70.88	71.24
SVM	82.01	88.26
Proposed method	90.79	95.03

**Table 6:** Vehicle detection results of different models.

Model	TPR (%)
Ref. [9]	81.92
Ref. [11]	88.61
Ref. [15]	90.27
Proposed method	96.49

## Data Availability

The data used to support the findings of this study are included within the article.
